The article "Formulation and Quality Control of Orally Disintegrating Tablets (ODTs): Recent Advances and Perspectives" was published in 2021. Journal: Biomed Res Int.

# Formulation and Quality Control of Orally Disintegrating Tablets (ODTs): Recent Advances and Perspectives

**DOI:** 10.1155/2021/6618934

**Published:** 2021-12-24

**Authors:** Mohammadali Poursharifi Ghourichay, Seyed Hossein Kiaie, Ali Nokhodchi, Yousef Javadzadeh

**Affiliations:** ^1^Department of Pharmaceutical Technology, Faculty of Pharmacy, Eastern Mediterranean University, Famagusta, Turkey; ^2^Student Research Committee, Tabriz University of Medical Sciences, Tabriz, Iran; ^3^Nano Drug Delivery Research Center, Kermanshah University of Medical Sciences, Kermanshah, Iran; ^4^Pharmaceutics Research Laboratory, School of Life Sciences, University of Sussex, Brighton, UK; ^5^Biotechnology Research Center and Faculty of Pharmacy, Tabriz University of Medical Science, Tabriz, Iran

## Abstract

Orally disintegrating tablets (ODTs) rapidly disintegrate or dissolve in the oral cavity without using water. Demand for ODTs has increased, and the field has overgrown in the pharmaceutical industry and academia. It is reported that ODTs have several advantages over other conventional tablets. Since some of them are absorbed from the mouth, pharynx, and esophagus as the saliva passes down into the stomach, in such cases, the bioavailability of the drug improves meaningfully. Furthermore, the immediate release property of ODTs makes them a popular oral dosage form in patients with swallowing challenges, children, and for cases with a need for rapid onset of action. The current review article explains the features of active ingredients and excipients used in the formulation of ODTs, discusses multiple ODT formulation and preparation techniques with their merits and demerits, and also, offers remedies for problems associated with ODTs. Moreover, quality control steps and required considerations are presented.

## 1. Introduction

Oral administration is the most widely used and convenient route with high stability and a small packaging size [1, 2]. The orally disintegrating tablet (ODT), as a delivery system, rapidly disintegrates in the mouth upon contact with saliva; therefore, it does not need additional water. It is available for absorption through pregastric mucosa. Mouth dissolving/disintegrating tablets (MDTs), quick disintegrating tablets, fast/rapid dissolving or disintegrating tablets (FDTs), quick/rapid melt tablets, orodispersible tablets, and porous tablets are the other recorded names for this type of dosage form [3, 4]. The need for rapid disintegration, rapid onset of action, and patient compliance, especially for pediatric, geriatric, psychiatric, paralyzed, and bedridden patients, leads to the emergence of OTDs in the 1980s [5] and the first articles on the formulation of ODTs using cellulose derivatives published by Watanabe et al. in 1995 [6].

The article "Formulation and Quality Control of Orally Disintegrating Tablets (ODTs): Recent Advances and Perspectives" was published in 2021. Journal: Biomed Res Int.

Food and Drug Administration (FDA) defines ODTs as “a solid dosage form containing medicinal substances which disintegrate rapidly, usually within a matter of seconds, when placed upon the tongue”. In comparison, European Pharmacopoeia (Ph. Eur.) defines them as “uncoated tablets intended to be placed in the mouth where they disperse rapidly before being swallowed and as tablets which should disintegrate within 3 min” [7]. Although ODTs are mentioned in some United States Pharmacopoeia (USP) monographs, it does not have such definitions for ODTs. According to the literature, ODTs have the merits of both liquids and conventional tablets. They are convenient with the short onset of action since they get absorbed through pregastric mucosa within seconds after administration [8]. For instance, ondansetron ODTs were applied for children without difficulties and reduced the occurrence of emesis. In addition, first-pass metabolism avoidance in ODTs has led to bioavailability enhancement which subsequently reduced dosing frequency and side effects [9]. It is reported that swallowing difficulty (dysphasia) due to diseases like motion sickness and allergic attacks may cause noncompliance and ineffective therapy. In these cases, comfort and quality of life will be enhanced via ODTs. Low-cost treatment is another upside of ODTs. The statistical evaluations revealed that olanzapine and risperidone ODTs were cheaper and more efficient than standard oral tablets (SOT) in schizophrenia [10]. Also, aripiprazole ODTs were more cost-effective than aripiprazole SOTs and olanzapine SOTs for schizophrenia patients in China [11]. Moreover, patients administering multidrug therapy can take the most advantages of fixed-dose combination (FDC)-ODTs. ODTs containing mitiglinide, voglibose, and mitiglinide/voglibose can be mentioned as examples; a most recent independent clinical trial with 13 healthy subjects indicated ease of FDC-ODT intake, unlike individual components-ODTs [12].

Although ODTs own several merits, they are still a niche product in the market as they have additional requirements. Taste perception is an important issue to consider; formulation of bitter drugs as ODTs is challenging, and taste masking materials should be employed [8], since they are compressed with a low force and possess a porous matrix [2, 13]. Therefore, handling friable and brittle ODTs is challenging. Hygroscopic characteristics and thermal and humidity sensitivity of ODTs can influence their physical integrity and lead to stability problems. Hence, using special materials is essential for their packaging.

The article "Formulation and Quality Control of Orally Disintegrating Tablets (ODTs): Recent Advances and Perspectives" was published in 2021. Journal: Biomed Res Int.

Moreover, decreased amount of saliva in patients on anticholinergic medicines may affect bioavailability [14]. There is a restriction on drug load in ODT minitablets (ODMTs) since the ODMTs may weigh just 6 mg [15]. Therefore, the preparation of high-dose substances like antibiotics is complex [16]. Environmental pollution and toxicity risks are two other drawbacks related to OTDs' preparation methods. In the coating technique, organic solvents dissolve polymers, and organic solvents are connected with toxicity risk, and solvent removal during the drying process is time-consuming [17]. In this review article, the features of active ingredients and excipients used in the formulation of ODTs were explained. In addition, the manufacturing method of multiple ODT formulations with their pros and cons alongside solutions for associated problems with ODTs were discussed in detail. The depicted quality control steps with required considerations were also discussed.

## 2. Features of APIs and Excipients

Most APIs used in ODT formulations have systematic effects rather than local effects. Drug and excipient properties should not affect tablet properties considerably; some characteristics like solubility, crystal morphology, particle size, hygroscopicity, and compressibility of a drug can change final ODT features. Analgesics, antihypertensives, anti-inflammatories, antibacterials, antifungals, and antilipidemics are the most prevalent substances formulated as ODTs [18]. The list of commercial ODTs is summarized in Table 1 [19]. There are several criteria for a drug used in ODT formulation that can make ODTs an acceptable and ideal dosage form. For example, the drug should be ionized, dispersed, and penetrated in mucosa without leaving any residue in the mouth cavity. Furthermore, the molecular weight of the API should be less than 500 Da. The active ingredient should be less than 50 mg for frequent use, with a short half-life, pleasant taste, and smell. Resistance to harsh environmental conditions, low cost of production, and is well-matched with existing processing, and packaging procedures make them even more appealing to patients and industry [20, 21].

As excipients also have a crucial role in ODT formulation, therefore, they should fulfil particular requirements, such as water solubility, pleasant taste, sweetness, and rapid dispersibility [22]. Some processed excipients like Ludiflash, Pharmaburst, F-melt, and modified chitosan are introduced to improve formulations, decrease wastage of material, and tackle problems such as compressibility, hygroscopicity, flowability, palatability, dissolution, and disintegration. These excipients are designed by the SeDeM expert system which includes several parameters in assessing excipients to attain a suitable powder characteristic prior to compression [23, 24]. Excipients like mannitol are used as diluents, but its modified type has many other valuable characteristics like higher stability, increased total surface size, and larger pore size that finally lead to a cost-effective product [25]. Excipients needed for an OTD preparation are listed in Table 2 with their role in the formulation. Ion exchange resins (indion 414/234, tulsion 234/344, and amberlite IPR 88) and gas evolving disintegrants (citric acid, tartaric acid, and sodium bicarbonate) are in the category of superdisintegrants. Among those disintegrants, sodium starch glycolate possesses good flowability, and cross povidone is fibrous and highly compactable. Sugar and sugar-based derivatives with high aqueous solubility and sweetness are used as bulking agents and sweeteners.

The article "Formulation and Quality Control of Orally Disintegrating Tablets (ODTs): Recent Advances and Perspectives" was published in 2021. Journal: Biomed Res Int.

It should be mentioned that before formulation, the safety of excipients should be assessed through guidelines such as International Conference on Harmonization (ICH), European Medicines Agency (EMA), Committee for Human Medicinal Products (CHMP), European Food Safety Authority (EFSA), The Joint FAO/WHO Expert Committee on Food Additives (JECFA), and indexed literature [26, 27].

Additionally, drug-excipient compatibility should be investigated prior to the selection of excipients. Physical, chemical, and biopharmaceutical interactions are considered as the potential interactions between API and excipient. Premature breakdown of enteric coat, interactions due to adjunct therapy (like complex formation between tetracycline and calcium), and increased gastrointestinal motility (because of sorbitol and xylitol) could happen due to unsuitable selection of excipients. Several thermal and nonthermal analysis methods and softwares for incompatibility evaluations are developed, which can further help in proper dosage form preparation [28].

## 3. Formulation Methods: Merits and Demerits

Molding, mass extrusion, sublimation, spray-drying, direct compression, and lyophilization (freeze-drying) which are commonly used to prepare ODTs are summarized in this review article (Figure 1). Their advantages and drawbacks are also presented in the current article. Additionally, there is also a wide range of patented techniques, including Wowtab®, Orasolv®, Fashtab® and Durasolv®, Zydis®, Durasolv®, Flashdose®, and Oraquick®, which have been reviewed by Tansel Comoglu & Emine Dilek Ozyilmaz [8].

### 3.1. Molding

ODTs prepared by molding technique disintegrate within 5 to 15 seconds. Molding or solid dispersion could be categorized into two groups as heat molding and compression molding. A molten mass containing a dispersed or dissolved drug is used to make molded tablets [32]. First, suspension of the drug with water-soluble sugars such as mannitol, lactose, sucrose, glucose, sorbitol or xylitol, and agar is prepared. These sugars act as a binder, also their presence creates a good mouthfeel. Then, the suspension is dispensed into blister packaging and molds, followed by evaporation of the solvent under vacuum conditions at 30°C which solidifies the agar solution and creates ODTs. In compression molding, powder blend is mixed with a hydroalcoholic solvent, then compressed into mold plates by implementing a low force, following that they let the tablets air-dried to lose their solvent and create a porous structure with high disintegration and dissolution rates. Valdecoxib and perphenazine ODTs are prepared via this method [33, 34]. The main disadvantages of this technique are high production cost and low mechanical strength, which leads to the breakage of ODTs through handling or when blister packs are opened. Adding binders like acacia, polyvinylpyrrolidone, and PEG may be helpful to overcome this drawback [35, 36].

The article "Formulation and Quality Control of Orally Disintegrating Tablets (ODTs): Recent Advances and Perspectives" was published in 2021. Journal: Biomed Res Int.

### 3.2. Mass Extrusion

In the mass extrusion process, water-soluble solvents such as PEG and methanol or ethanol are used to soften the powder mixture. Then, it is sieved through the extruder or syringed. After extrusion, alcohol was removed by evaporation. A solidified string shaped gel is resulted, which subsequently crushed into granules using a mortar. Then, these granules could be mixed with other ingredients and turned to ODTs via compaction methods discussed in the following sections [37]. In mass extrusion, PEG stearate is implemented as a binder to improve physical strength and disintegration. Through this technique masking the bitter taste of the drug is possible by coating granules using compounds like Eudragit E 100, ethylcellulose, hydroxypropyl methylcellulose (HPMC), hydroxypropyl cellulose (HPC), polyvinyl alcohol, and polyvinyl acetate [38].

### 3.3. Spray-Drying

Generally, in the spray-drying method, solid dispersions and micronized particles of drug/excipients are prepared for oral or inhalation administration [39]. First, a liquid mixture of material is sprayed into a hot chamber to obtain a highly porous structure. Then, typically, these microparticles were mixed with mannitol and kneaded with distilled water before drying at 60°C for 2 h. After that, the prepared granules were sieved and blended with other excipients and finally compressed into tablets using the compaction methods discussed in the following sections. Tablets prepared by this method possess high porosity and disintegrate rapidly in the mouth. The significant disadvantages of this method are the high cost of production and fragility of the product, which makes conventional packing methods inappropriate for this dosage form.

The article "Formulation and Quality Control of Orally Disintegrating Tablets (ODTs): Recent Advances and Perspectives" was published in 2021. Journal: Biomed Res Int.

### 3.4. Cotton-Candy Process

This process implements a distinctive spinning instrument to yield crystalline flosses. A candy floss matrix results from simultaneous flash melting and spinning of saccharides or polysaccharides like polymaltodextrin and polydextrose using proper flow at 180–266°C. Next, the prepared matrix gets milled and blended with API/excipients and compressed into ODTs. This routine is specially implemented for covering the bitter taste of drugs. Additionally, partially, recrystallization of the candy floss matrix may improve the flow properties, compressibility, and mechanical strength. Also, it causes the accumulation of a large amount of drugs, but it is not suitable for thermo-labile drugs [19].

### 3.5. Lyophilization (Freeze-Drying)

Lyophilization is a procedure in which drying of thermo-sensitive APIs happens under a low temperature by applying a vacuum. Freeze-dried ODTs are often called lyophilizates. Usually, they are very light, with highly porous structures and disintegrate fast. Formulating freeze-dried OTDs in a liquid state leads to accurate dosing. Furthermore, handling potent or toxic APIs in a liquid state is safer for operators than dusty powder. However, the process is pretty pricy and unsuitable for formulations which are not stable at high temperature and humidity [13, 40].

Zydis and Lyoc are two lyophilization platforms. Zydis process starts with forming an aqueous bulk liquid constituted of gelatin as polymeric binder and mannitol as a mechanical booster. Gelatin acts as a glue to retain API and filler particles together in the final ODT. Furthermore, the presence of a hydrophilic filler (highly soluble in water) such as mannitol can promote disintegration [41]. Additionally, colorants, pH modifiers, taste-masking agents, and preservatives can be added to the formulation. In the following step, the liquid formulation is poured into blister pockets and hastily frozen using a tunnel freezer. After complete freezing, blisters are conveyed to large industrial batch freeze-dryers for primary and secondary drying under a vacuum. After drying, blisters are airtight and packed. In this platform, the drug is low dose and water-insoluble with a small particle size to decrease the processing time and achieve a smooth mouthfeel.

Zydis has some limitations; firstly, inconstant hardening time in the semicontinuous freezing mode leads to intrabatch pore-size variability [42]. Secondly, some people have ethical constraints for animal products like gelatin; also, gelatin has inconsistent quality, and its viscosity depends on temperature, pH, and time [2]. Polyvinyl alcohol (PVA) was examined and reported as a substitute for gelatin. Xanthan gum was picked as a viscosity booster if PVA does not inhibit drug sedimentation throughout the preliminary freeze-drying process. Sedimentation could be measured using raman spectroscopy and reduced by regulating the xanthan gum concentration [2]. Polymers such as gelatin, dextran, and alginate are necessary for the glassy amorphous structure to provide stability and flexibility during manufacturing. For example, in terbutaline sulfate ODT preparation, gelatin and sodium alginate have opted as a matrix former, and sodium alginate was also used as a viscosity modifier. Mannitol that gives crystallinity and hardness to freeze-dried ODTs was used as a filler; PEG 4000 (as disintegration accelerator), pluronic F68 (as a surfactant to improve low solubility of TBS), and hydroxypropyl methylcellulose were also added to the formulation. In addition, simethicone was selected as an antifoaming agent to obtain uniform ODTs since foaming in the mixing process may cause shape variation [26].

The article "Formulation and Quality Control of Orally Disintegrating Tablets (ODTs): Recent Advances and Perspectives" was published in 2021. Journal: Biomed Res Int.

In Lyoc technology, an oil-in-water emulsion is prepared using water-soluble fillers such as mannitol or lactose. Usage of a large amount of fillers leads to a paste-like form which finally prevents sedimentation in the formulation. Then, like Zydis process, freeze-drying phases happen in commercial freeze-dryers [43]. Low-porous particles and higher drying time made the Lyoc strategy less economical.

### 3.6. Compaction Methods

In this process, a compression device promotes agglomeration and bonding of particles by applying pressure and prepares integral structures like tablets or briquettes. The applied compression force depends on tablet size, APIs, and excipient properties. For example, according to Stoltenberg and Breitkreutz's study, in the formulation of ODMTs, compression force should be in the range of 3 to 8 kN [44]. The choice of excipient is another vital factor since compression lessens the porosity of the product, which is crucial for a fast disintegration; this matter necessitates the addition of superdisintegrates and sugar-based fillers [40, 45]. The compaction process ranges from confined compression devices such as tabletting to serial devices like extrusion. The following techniques are based on the compaction approach.

#### 3.6.1. Sublimation

In sublimation technique, drugs and a swiftly volatilized element like urea, camphor, menthol, ammonium carbonate, ammonium bicarbonate, benzoic acid, hexamethonium tetramine, naphthalene, phthalic anhydride, and urethane were used along with other excipients. Solvents such as cyclohexane/benzene were occasionally used for further augmentation of porosity [46, 47]. The prepared blend is compressed as a tablet form; then, the volatile material is evaporated via pressure and temperature, which causes that the residual bulk becomes porous. High porosity is the essential characteristic of tablets prepared by the sublimation method. Additionally, volatilization of volatile material eliminates the complexity of processes such as the sublimation of frozen water [48]. Captopril, an angiotensin-converting enzyme inhibitor, is used to manage emergency hypertension, and it is projected to provide maximum pharmacological effect within 1-2 h after oral administration. The need to provide captopril tablets for patients with swallowing problems makes captopril a good candidate for ODT formulation. Captopril ODTs prepared by this method have been studied *in vitro* and *in vivo*. In a recent study, captopril ODTs formulated using 5% croscarmellose sodium (Ac-di-sol®) and 10% camphor revealed appropriate rigidity, shortest disintegration time (3.425 ± 0.12 kilopond, 17.48 ± 1.36 s), and highest in-vitro drug release (99.51 ± 0.24%) after 8 min. Furthermore, the *in vivo* assessment showed 15 min faster stabilization of mean arterial pressure in hypertensive rats [9].

The article "Formulation and Quality Control of Orally Disintegrating Tablets (ODTs): Recent Advances and Perspectives" was published in 2021. Journal: Biomed Res Int.

Salbutamol sulfate ODTs is the other OTD that has been prepared and evaluated by Suresh and Joshi [49] using the sublimation method. Adding camphor/ammonium bicarbonate to the formulation as a volatile substance improved the physicochemical properties of the ODT and led to disintegration within 5-40 s [49].

#### 3.6.2. Melt Granulation

In this process which does not require solvents or a drying process, a binding material with a low melting or softening point is used. Melted materials act as a binder and harden at room temperature to develop a solid dosage form. The waxy binder melts inside the mixer to prepare granules; then, granules get dried in tray dryers. After the sieving to acquire uniform granules, the granules are mixed with other ingredients and compressed into tablets. Particles manufactured by melt granulation are controlled-release and cost-effective. Hasian optimized process parameters to manufacture ODTs having melt adsorption-particles. They prepared melt adsorption particles with Neusilin US2 as the adsorbent. They used five hydrophobic materials including, glyceryl monostearate, stearic acid, glycerol fatty acid ester, microcrystalline wax, and hydrogenated castor oil to elect the most appropriate material for controlled release formulation. Finally, they introduced glycerol fatty acid ester as optimal wax due to its drug release profile and tabletability [17].

The article "Formulation and Quality Control of Orally Disintegrating Tablets (ODTs): Recent Advances and Perspectives" was published in 2021. Journal: Biomed Res Int.

#### 3.6.3. Crystalline Transition Process

It has been shown that the shift from the amorphous to the crystalline state via compressing two saccharides, one with high and the other with low compressibility index, could create ODT with suitable hardness [50]. Sucrose, lactose, glucose, xylitol, mannitol, and erythritol are recommended as low-compressible saccharides, maltose, sorbitol, trehalose, and maltitol as high-compressible saccharides [51]. Sugimoto et al. have used fluidized bed granulation for the crystalline transition process. They first granulated mannitol with sucrose aqueous solution in a fluidized bed granulator, followed by mixing the granules with magnesium stearate, and compressed the mixture into tablets with a diameter of 10 mm by a tabletting device. According to their result, an efficient ODT results from compressing mixture before the crystallizing process of the amorphous sucrose [52].

#### 3.6.4. Phase Transition

This route comprises compressing the powder including two sugar alcohol with high and low melting points and afterwards heating the compressed mass at the temperature amongst their melting points. Since the low compressibility and higher interparticular bonds decrease hardness, while after heating, the hardness improves because of diffusion and solidification of sugar alcohol, Kuno et al. used this method to manufacture ODTs [53]. In the phase transformation technique to maintain the porosity, a low compression force is followed by a humidity or heat treatment to increase mechanical strength, though humidity or heat implementation may lower the stability of water-sensitive or thermolabile drugs [54].

#### 3.6.5. Conventional Methods

Conventional methods such as wet granulation, dry granulation, and direct compression are used to prepare ODTs. Shanmugam has comprehensively reviewed granulation techniques [55], and it was pointed out that wet granulation is the commonly used method. Granules are manufactured by wet massing of the excipients and API by granulation liquid with or without binder, while dry granulation entails no liquid. ODT of glibenclamide is prepared by using the wet granulation technique [56].

Direct compression is the most straightforward approach to make tablets, particularly for large-scale ODT making. This routine contains superdisintegrants like crospovidone, croscarmellose, alginic acid, and calcium silicate. The direct compression method has been used to prepare tramadol hydrochloride OTDs. First, taste-masked granules of tramadol hydrochloride are prepared using Eudragit E100 via mass extrusion method, then OTDs are formulated using sodium starch glycolate, Ac-Di-Sol®, and crospovidone as the superdisintegrants. In this way, the rapid onset of action resulted in postoperative pain alleviation [38].

The article "Formulation and Quality Control of Orally Disintegrating Tablets (ODTs): Recent Advances and Perspectives" was published in 2021. Journal: Biomed Res Int.

Levodopa/benzyl hydrazine is another example of ODTs prepared by direct compression and provided ease of use for patients with Parkinson. Formulation with microcrystalline cellulose 25.7%, cross-polyvinylpyrrolidone 6.22%, sodium carboxymethyl starch 5.36%, and mannitol 22% led to shorter disintegration time and faster dissolution pattern [57]. Dosing of the formulation in direct compression can be pretty challenging. Also, the disintegration time of the ODTs could be affected by the amount and type of the binding agent and superdisintegrant. Moreover, the direct compression technique requires more effervescent agents [54]. To solve the drawbacks mentioned above, novel multichannel ODTs are designed. Multiple channels formed in the ODTs allow water to pierce the core and speed up disintegration [58]. Novel multichannel ODTs containing aripiprazole with accelerated tablet disintegration and lower costs were developed by wet compression methods and enhanced patient compliance [59].

## 4. Quality Control Tests for ODTs

ODTs' quality control tests are comparable to those of conventional tablets, except for minor dissimilarities. For instance, wetting time, water absorption ratio, moisture uptake, in vivo disintegration time, and taste evaluation are specifically used for ODTs. Quality control tests are allocated into two groups as precompression and postcompression tests.

### 4.1. Precompression Tests

Precompression tests, which include determining the angle of repose, bulk density, tapped density, Hausner ratio, and Carr's index [60], are implemented on the mixture of powder that is used for ODT manufacturing. The purpose of precompression studies is to ensure that powder has the desired characteristic for subsequent processing.

The angle of repose demonstrates frictional force in a loose powder. When the angle is lower than 30 for a given powder, it represents free-flowing behavior. The flow tendency and compressibility are depicted by Hausner ratio and Carr's index, respectively. Accordingly, when Hausner ratio is lower than 1.25, flowability is good, while excellent compressibility is seen for Carr's index less than 15 [60]. As bulk density is directly related to particle size and the adhesion tendency, hence, it is helpful for a selection of packing materials and transportation considerations.

### 4.2. Postcompression Tests

Postcompression tests are implemented on the ultimate ODTs. These tests as mentioned in Table 3 include determining weight variations, hardness, thickness, friability, wetting time, water absorption ratio, and moister uptake. In vitro and in vivo disintegration time, taste evaluations, and dissolution tests are also in the postcompression test category, which is summarized below.

The article "Formulation and Quality Control of Orally Disintegrating Tablets (ODTs): Recent Advances and Perspectives" was published in 2021. Journal: Biomed Res Int.

#### 4.2.1. In Vitro Methods for Determining Disintegration Time

ODTs must be crumbled easily to be dispersed in the patient mouth salvia. Besides, they need to be durable enough to bear the mechanical pressure of production and transportation. To determine this quality, a disintegration time test needs to be done both in in vitro and in vivo environments [61].

In vitro disintegration time tests have been thoroughly reviewed by Ölmez, and Vural [16]. They have mentioned Ph. Eur. methodology, texture analysis method, charge-coupled device (CCD) camera method, rotary shaft method, and a modified USP method as five determining tests of the start and endpoints of disintegration. Also, in a recent study Koner et al., they have introduced the Aston test as a novel disintegration method that can mimic the environment of the oral cavity [61]. In their study, they compared their system with the USP method. They exhibited that the Aston test was able to discriminate between different ODTs with narrow disintegration time windows, as well as between immediate-release tablets and ODTs. It also demonstrated a linear in vitro/in vivo correlation (IVIVC) in comparison with a “hockey stick” profile of the USP test. Overall, they concluded that their test is a robust method for assessing ODT disintegration time in the pharmaceutics and monitoring authorities [61].

According to Ph. Eur, single ODT was placed into three of the six cylinders of the basket-rack assembly. Then, this apparatus oscillated 31 cycles per minute in a 900 mL water bath at 37°C. The time for the disintegration of each tablet is recorded, and each ODT type must completely disintegrate within 3 minutes to be considered a pass [62]. Similarly, in the modified USP dissolution test, tablets are placed and suspended in the middle of the container of USP apparatus II (100 rpm, 900 mL, 37°C). The time needed for whole tablet disintegration and passing through sinker's sieve was considered as disintegration time [63]. The process in a texture analysis method is different; in this analysis device, a tablet adheres under a probe; afterwards, it is pushed towards the base of the beaker containing distilled water by a stable pressure, and the extent of penetration is measured [64]. The rotary shaft method is a reminiscent texture analysis technique. In this test, ODT is placed on a perforated plate, and the rotary shaft applies mechanical stress. Then, an electrical sensor determines the end of disintegration [65].

The article "Formulation and Quality Control of Orally Disintegrating Tablets (ODTs): Recent Advances and Perspectives" was published in 2021. Journal: Biomed Res Int.

In a CCD camera method, the temperature is delicately adjusted, by two steel containers, an internal container with a capacity of 200 mL distilled water and the external container as a thermostat. CCD camera takes pictures and transfers them to a computer equipped with motion capture followed by calculating the disintegration time using image analysis software. In this method, differentiation of minor distinctions among different ODT formulations is possible since disintegration occurs in a mildly agitated medium. In addition, it provides qualitative information like morphological changes in the tablet during disintegration [66].

As mentioned earlier, the recently established Aston test has been made to mimic conditions of the oral cavity. To mimic the in vivo situation, the temperature (37 ± 1°C) and relative humidity (93 ± 3%RH) of the test is set up by a hot plate and potassium chloride. A slightly flattened silicone pipe with 4 mm holes is used as a disintegration bed. A flow of water (10 ml/min) through the holes simulated saliva and the interaction of media with the tablet lead to disintegration, which subsequently is measured by a texture analyzer [67]. Each test was repeated eight times, and disintegration time was calculated by the plot of distance/time [61].

#### 4.2.2. In Vivo Determination of Disintegration Time, Taste, and Mouthfeel

Besides the in vitro disintegration test, in vivo disintegration and taste evaluation are also performed on ODT [68]. In vivo determination of disintegration time may be carried out with randomly chosen healthy volunteers. First, volunteers are asked to wash their mouths. A tablet is put on their tongue, and the time until the disintegration of the last granule will be measured. If tablets contain active substances with side effects on healthy volunteers, prior permission must be acquired from the Board of Ethics.

Taste masking is an essential step in the formulation of drugs with bitter taste; otherwise, patient compliance might be a challenge. Adding sweeteners like sugar is the most common way to eliminate the bitter taste. Adjusting the pH is recommended as another useful technique [69]. When these methods could not improve the taste, adding physical barriers like surrounding the API particle by coating or inclusion of them inside the compounds like cyclodextrin could be employed to reduce the contact between the API and taste buds [70, 71]. The application of coating material requires careful consideration since it may alter drug's biopharmaceutical behavior [72]. Preparation of solid dispersions, hot-melt extrusion, and using nanotechnology are additional formulation techniques that increase solubility besides taste-masking [73–75].

The article "Formulation and Quality Control of Orally Disintegrating Tablets (ODTs): Recent Advances and Perspectives" was published in 2021. Journal: Biomed Res Int.

For taste and mouthfeel, according to the taste and grittiness evaluation protocols, six or twelve volunteers are requested to report their immediate judgments after the tablet is placed in their tongue and after 3-4 min. In vivo taste assessment of ODTs used in pediatric is a bit challenging since the perception of adults and children may differ dramatically [27]. The taste and mouthfeel are valued in a range of 1 to 5. Each test needs to be repeated in triplicate with an interval of 15 minutes. In evaluations, 1 is considered as no roughness and no bitterness; 2 equals slight roughness and no bitterness; 3 means there is roughness but no bitterness; 4 is appreciable roughness and bitterness while 5 is an indication of strong roughness and appreciable bitterness [57].

#### 4.2.3. Dissolution Test

USP apparatus 1 or 2 can be implemented for dissolution examinations. When apparatus type 1 (basket method) is used, some errors could occur due to the obstruction of basket pores by clog forming; therefore, in these cases, apparatus type 2 (paddle method) is used. The preferred rotation speed is 50 rpm for the dissolution test, but the rotation speed can be 100 rpm for the taste-masked ODTs. it should be kept in mind that a low paddle speed could create better discrimination between in vitro dissolution profiles. According to FDA, a minimum of 85% of the API in ODTs ought to be dissolved in 30 min to meet the requirement. Analytical methods such as UV-Vis spectroscopy and high-pressure liquid chromatography (HPLC) are generally used to measure the quantity of dissolved API [76].

## 5. Packaging Considerations

Packing is one of the essential steps in ODT development. As excipients used in the formulation of ODTs should disintegrate/dissolve in a minimum amount of water, and also, they may attract moisture from the surrounding; therefore, special consideration is needed for their storage like a dry place. In addition, ODTs prepared by diverse techniques have different mechanical strengths; therefore, they need distinct packing [81]. For example, ODTs designed by Zydis are porous and have less physical resistance and sensitivity to moisture.

In an accelerated stability study, the effect of three types of packaging and excipient were investigated [76]. According to the report, the presence of StarLac® as filler/binder in ODT formulations limited the moisture absorption, and it was independent of the packaging material. While the replacement of StarLac® with polyols caused an increase in the weight of tablets. The weight gain was dependent on the packaging material. For instance, it was shown that the highest increase in weight was observed for the polyvinylidene chloride/aluminium blister (PVDC) blister whereas for tablets packed in the amber glass bottles with plastic cap weight change was not dramatic [82].

The article "Formulation and Quality Control of Orally Disintegrating Tablets (ODTs): Recent Advances and Perspectives" was published in 2021. Journal: Biomed Res Int.

## 6. Accelerated Stability Studies

In the accelerated stability test according to ICH guidelines, 20 tablets are packed in each 10 mL high-density polyethylene (HDPE) bottle and sealed thermally, then placed in a humidity chamber (45 ± 2°C and 75% ± 5% RH), up to 3 months. At the end of each month, postcompression tests are carried out on samples. Passing the stability test means no significant differences between postcompression studies of initial and accelerated stability samples [79, 83, 84].

## 7. Conclusion and Perspective

ODTs have several positive aspects compared with the other oral dosage forms. They offer low-cost treatment with improved bioavailability, efficacy, and patient compliance. They are also suitable for pediatric and geriatrics use and patients with dysphasia or parlayed psychiatric and bedridden patients. However, there are bottlenecks in their manufacturing and storage; for instance, ODTs may attract water from the surrounding since excipients used in the formulation can disintegrate in minimum water. In addition, some people have ethical constraints for animal products like gelatin. Moreover, bitterness which may remain in the mouth after swallowing the saliva due to ineffective taste masking affects patient's compliance. Dosing of the formulation in the direct compression and more effervescent usage are other challenges ahead of the formulation. Additionally, the development of ODTs with lipophilic API is complicated, and environmental pollution and toxicity risks are two other drawbacks related to OTDs' preparation methods.

With the recent developments in the pharmaceutical sciences, limitations like short half-life have been solved. ODTs with controlled release properties such as Cotempla XR-ODT™, Adzenys XR-ODT™ as extended-release forms, and Dexilant® as the only dual delayed-release could be mentioned as examples. However, according to the data in Table 1, there are not many delayed-release and multiple-dose ODTs in the market.

Novel multichannel ODTs which allow water to penetrate the core have solved the disintegration problem. Sublimation and melt granulation methods which do not require solvents may help tackle environmental issues. Besides, particles manufactured by melt granulation are controlled-release and cost-effective.

Last but not least, new techniques such as the Aston test which was able to distinguish different ODTs with narrow disintegration time windows, as well as between immediate-release tablets and ODTs, have paved the way for evaluating ODT formulation. However, there are still some unsolved problems, and it is hoped that recent advances in formulation technology and the emergence of excipients like Ludiflash, Pharmaburst, F-melt, and modified chitosan would help overcome some of the limitations.

The article "Formulation and Quality Control of Orally Disintegrating Tablets (ODTs): Recent Advances and Perspectives" was published in 2021. Journal: Biomed Res Int.

## Figures and Tables

**Figure 1:** ODT formulation techniques.

**Table 1:** Commercial ODT formulations on the market.

Product	Active substance	Company
Benadryl®	Diphenhydramine	Yamanouchi/Pfizer, Morris Plains, NJ, USA
Claritin® RediTabs®	Loratadine	R.P.Scherer/Schering-Plough, Kenilworth, NJ, USA
Alavert®	Loratadine	CIMA/Wyeth Consumer Health, Madison, NJ, USA
Zomig®	Zolmitriptan	CIMA/Astra Zeneca, Wilmington, DE, USA
Tempra®	Acetaminophen	CIMA/Mead Johnson, Chicago, IL, USA
NuLev.	Hyoscyamine	CIMA/Schwarz Pharma, Milwaukee, WI, USA
Ultram®	Tramadol	JANSSEN PHARMS
Excedrin®	Acetaminophen, aspirin	Ethypharm/BMS, Philadelphia, PA, USA
Maxalt®	Rizatriptan	R.P.Scherer/Merck, Kenilworth, NJ, USA
Zyprexa®	Olanzapine	R.P.Scherer/Eli Lilly, Indianapolis, USA
Pepcid RPD	Famotidine	Merck and Co., NJ, USA
Zofran®	Ondansetron	R.P.Scherer/Glaxo SmithKline, Philadelphia, PA, USA
Feldene	Piroxicam	Pfizer Inc., NY, USA
Risperdal®	Risperidone	Janssen Pharmaceuticals, Beerse, Belgium
Remeron®	Mirtazapine	CIMA/Organon, Oss, Netherlands
Triaminic®SoftChews®	Phenylephrine-dextromethorphan	CIMA/Novartis Consumer Health, Basel, Switzerland
Zelapar ™	Selegiline	Amarin Corp., London, UK
Nimulid-MD	Nimesulide	Panacea Biotech, New Delhi, India
Romilast	Montelukast	Ranbaxy Labs Ltd., New Delhi, India
Torrox MT	Rofecoxib	Torrent Pharmaceuticals, Ahmedabad, India
Olanex Instab	Olanzapine	Ranbaxy Labs Ltd., New Delhi, India
Mosid-MT	Mosapride citrate	Torrent Pharmaceuticals, Ahmedabad, India
Febrectal	Paracetamol	Prographarm, France
Adzenys XR-ODT™	Amphetamine (extended-release)	Neos Therapeutics
Ambien®	Zolpidem (extended-release)	Sanofi Aventis
Cotempla XR-ODT™	Methylphenidate (extended-release)	Neos Therapeutics
Dexilant®	Dexlansoprazole (only dual delayed-release)	Takeda, Lexington, MA, USA

**Table 2:** Approved excipients used in ODT formulation.

Ingredient type	Example	Role	Ref.
Superdisintegrant	Crospovidone, croscarmellose sodium, sodium starch glycolate, sodium carboxymethyl cellulose, microcrystalline cellulose, spray-dried lactose, acrylic acid, alginic acid, sodium alginate, soy polysaccharides, Isphagula husk pregelatinized starch, modified corn starch, ion exchange resins, gas evolving disintegrants	(i) Burst disintegration facilitator	[4]

Bulking material	Sugar and sugar-based derivatives (dextrose, fructose, isomalt, lactilol, maltitol, maltose, mannitol, sorbitol, starch hydrolysate, polydextrose, and xylitol)	(i) Textural properties (disintegration time) improver	[29]

Emulsifier	Alkyl sulfates, propylene glycol, lecithin, sucrose esters, sodiumdoecylsulfate, sodium lauryl sulfate, polyoxyethylene sorbitan fatty acid esters (Tweens)	(i) Disintegration accelerator (ii) Bioavailability enhancer of immiscible substances	[30]

Sweetener	Sodium saccharin, sugar alcohols, natural sugars (sugar, dextrose, fructose), sugars derivatives, aspartame, vanilla, bubble gum, grapefruit	(i) Bitter taste mask (ii) Tablets' acceptability enhancer	[22]
Flavor	Peppermint flavor, clove oil, bay oil, anise oil, eucalyptus oil, thyme oil, oil of bitter almonds, vanilla, citrus oils, fruit essences	(i) Patient compliance and acceptability improver	[31]

The article "Formulation and Quality Control of Orally Disintegrating Tablets (ODTs): Recent Advances and Perspectives" was published in 2021. Journal: Biomed Res Int.

**Table 3:** Postcompressing tests of ODTs.

Parameters	Properties	Purpose and considerations		Ref.
Weight variation	The weight of 20 randomly chosen tablets is determined then the mean weight is calculated	Weight average (mg)	Max SD.	[77]
		130 or <130	10	
		130-324	7.5	
		324 or >324	5	

Content-uniformity	3 tablets of each formulation were powdered and then the UV absorbance of mixture equivalent to 1 mg of API is measured	If the API is less than 25 mg, the content-uniformity test is used. Otherwise, the weight-variation test is applicable		[78, 79]

Hardness	By using a Varian tablet hardness tester crushing strengths of six randomly selected tablets were measured and expressed in Newton units	It shows the mechanical integrity of tablets		[73, 77]

Porosity	It is measured by a mercury porosimeter	Porosity moderately shows the amount of water penetration to formulation and disintegration time		[61]

Thickness and diameter	Diameter and thickness of ten randomly selected tablets were measured by putting between the arms of the digital Vernier caliper and recorded as average diameter and thickness	—		[68, 73]

Friability	Some tablets are weighed (initial weight) before putting them into the friabilator (at 25 rpm and 4 min), then after weight loss measurement, the friability value is calculated	According to USP 24: % friability value should be <1		[79]

Wetting time/water absorption ratio	10 mL of eosin solution is poured into a dish and weight of tablets before placing in the dish and after reaching the eosin to the upper part of them is measured	Short wetting time leads to fast disintegration		[68]

Moisture uptake	10 tablets are put in a desiccator (37°C, 1 d), then tablets are weighed and exposed to 75% RH (25°C, 15d) and increase in weight is recorded	Used to evaluate the stability of the formulations		[80]

RH: relative humidity.
